# Effects of Nutritious Meal Combined with Online Publicity and Education on Postoperative Nutrition and Psychological State in Patients with Low Rectal Cancer After Colostomy

**DOI:** 10.1155/2022/1541385

**Published:** 2022-06-28

**Authors:** Lijuan Qu, Mei Zhou, Yi Yu, Kaili Li

**Affiliations:** ^1^Department of Gastrointestinal Surgery, The Affiliated Hospital of Qingdao University, Qingdao, 266000 Shandong, China; ^2^Department of Wound Stoma Clinic, Laixi People's Hospital, Qingdao, 266600 Shandong, China; ^3^Department of Thoracic Surgery, The Affiliated Hospital of Qingdao University, Qingdao, 266000 Shandong, China; ^4^Department of Gastrointestinal Surgery Ward, Jinan 4th People's Hospital, Jinan, 250031 Shandong, China

## Abstract

**Objective:**

To investigate the effects of nutritious meal combined with online publicity and education on postoperative nutrition and psychological state in patients with low rectal cancer after colostomy.

**Methods:**

The clinic data of 88 patients with low rectal cancer who received the colostomy in our hospital (August 2020-August 2021) were retrospectively reviewed. Among them, 44 patients received nutritious meal combined with online publicity and education and they made up the study group, and the others were given conventional care and they made up the reference group. The nutrition indicators, scores of the World Health Organization Quality of Life (WHOQOL)-BREF, and other materials of the patients in the two groups were compared.

**Results:**

After intervention, the various nutrition indicators, immune indexes, and WHOQOL-BREF score of the study group were all prominently higher than those of the reference group (*P* < 0.001). Compared with the reference group, the study group after intervention achieved markedly lower self-rating anxiety scale (SAS) score and self-rating depression scale (SDS) score (*P* < 0.001) and obviously lower total incidence of complications (*P* < 0.05).

**Conclusion:**

Combining nutritious meal with online publicity and education can effectively improve the postoperative nutrition and immune function of the patients with low rectal cancer after colostomy, and this intervention contributes to releasing the patients' adverse emotions. Further study helps to provide these patients with favorable solutions.

## 1. Introduction

Low rectal cancer, as a kind of common malignant tumor in clinic, refers to the rectal cancer occurring less than 8 centimeters from the anal verge [1, 2]. Colostomy is the common treatment for this cancer at present. It is difficult to preserve the anus and the function of anus during the surgery due to the anatomical location, so the permanent colon stoma is made on the abdominal wall to replace the anus to perform the defecate function [3]. However, the patients with the stoma cannot control the defecation at their willing, leaving inconvenience to their life and reducing their physiological and psychological adaptation. According to relevant studies [4], because of the particular structure of the rectum and the tumor consumption, as well as the surgical trauma, most patients suffer from nutrient intake disorder, which leads to the malnutrition, immunocompromise, and aggravated inflammation and is not conducive to the postoperative rehabilitation. In the past, parenteral nutrition treatment was mostly adopted in the clinic [5], but with the deepening of the studies on the clinical nutrition, it is found that parenteral nutrition treatment, with inadequate nutritional drugs, may lead to damages to the intestinal barrier and tissue atrophy of the intestinal mucosa in the long term. In recent years, the importance of nutritious meal in the comprehensive treatment during perioperative period has been gradually recognized [6]. Nutritious meal not only provides the nutrition support but also reduces the occurrence of postoperative complications to a certain extent and can effectively promote the recovery of gastrointestinal tract and other organ functions and improve patients' prognosis. Actually, its curative effects have been confirmed in the postoperative rehabilitation of the patients undergoing total resection of bladder tumor and oral cancer surgery[7, 8]. The patients with colostomy needs to experience a long rehabilitation period after the surgery, and the scientific publicity and education in clinic can provide guidance and assistance to the patients. As the intelligent publicity and education is continuously promoted, the online publicity and education have received more and more favor from the patients [9], and it has been applied to the breast cancer patients, the patients with osteoporotic lumbar compression fracture, and other patients. At present, there is no study reporting the value of nutritious meal combined with online publicity and education on the low rectal cancer. This study further summarizes the treatment methods in the clinic, so as to provide more theoretical and data support for the postoperative rehabilitation of the patients with low rectal cancer.

## 2. Materials and Methods

### 2.1. General Data

Eighty-eight patients with low rectal cancer who received the colostomy in our hospital (August 2020-August 2021) were selected as the research objects, and this study was conducted in accordance with *Declaration of Helsinki* (*2013*) [10]. The inclusion criteria were as follows. ① The patients met the diagnostic criteria in the National Comprehensive Cancer Network (NCCN) 2017 Version 1.0: Guideline for Colorectal Cancer [11], and their diagnoses were confirmed by proctoscopic examination and pathological biopsy. ② The Magnetic resonance imaging (MRI) and digital rectal examination indicated that the distance between the lower edge of the tumor and the anus was ≤8 centimeters. ③ The patients conformed to the treatment indication of the colostomy and were ≥18 years old. The exclusion criteria were as follows. ① The patients were complicated with severe cerebral, cardiac, liver, or renal dysfunction. ② The patients were complicated with other malignant tumor. ③ The patients suffered from the stenosis or perforation caused by the tumor, and they were under urgent need for surgical treatment. ④ The patients were in stage IV in term of the tumor staging before the surgery.

### 2.2. Methods

The reference group was given routine nursing after surgery. The primary nurses and the doctor jointly formulated nursing measures for the colon stoma and offered routine clinical education and publicity and nursing interventions. The clinical education and publicity included the following contents. The patients were informed of the causes and treatment of rectal cancer, the necessity of colostomy (in order to gain the patients' understanding), self-care methods for the colon stoma (including correct replacement of the colostomy bag and regularly cleaning the skin around the colon stoma), and relevant matters needing attention after the surgery. Besides, the patients were guided to keep reasonable and balanced diet and were recommended to have multiple meals with small amount for each and take less gas-producing foods. Also, they were encouraged to communicate more with their families [12].

The study group received nutritious meal combined with online education and publicity after surgery. The nutritious meal was prepared as below. Nutritious meals were developed, because oral feeding in the early stage after surgery simply could not meet the nutritious demand of the patients' body, so a nutritional supplement was given to the patients so as to increase the intake of protein and calories. Based on the specific situation, nutritious meals were prepared for the patients to supplement the energy needed, and normal oral feeding combined with oral nutritional supplement was adopted to meet the body's demand for protein and other energy. A personalized nutritious diet plan was established by the nutritionists according to the patients' clinical status to satisfy the nutritious supply. When preparing the nutritious meals, the nutritionists selected the most reasonable nutrition agents according to the patients' individual differences. The patients received the online publicity and education during the perioperative period, specifically as follows. ① the online publicity and education team was formed by an international enterostomal therapist, a senior nurse, and three nurses, with the senior nurse as the team leader, who was responsible for the daily management and supervision of the other members. All the team members had good communication and consultation ability (those with clear thinking, and ability to express their main thoughts and understand others' expressions), so as to enhance the strength of the whole team and provide adequate safeguard for the patients' postoperative recovery. The team members received training in the methods of online publicity and education, as well as relevant professional knowledge, and needed to pass the assessment before they were allowed to begin their work. ② The team leader set up the WeChat groups in advance to communicate with the patients or their families and to spread the health knowledge about colostomy. ③ The team members should keep good communication with the patients, and the enterostomal therapist provides the patients with the whole-course nursing (including psychological guidance, stoma location, responsibility nursing, health publicity, and education and dietary intervention) during their treatment in the hospital. Therefore, the team members should get familiar with the patients' condition and the local condition of the stoma and stress the importance and significance of the postoperative intervention. ④ Sending relevant contents to WeChat groups, the enterostomal therapist should find relevant knowledge of colon stoma and compose and timely send the message to the WeChat groups in the form of text, picture, audio, and video. On average, the enterostomal therapist sent the message two times a week for a month. The specific arrangements were as follows. In the first week, the patients were given psychological counseling and were informed of the correct methods for replacing the colostomy bag. In the second week, the patients were guided to pay attention to and prevent the complications of stoma, and to observe the defecation, the abdomen, the skin around stoma, and the local condition of stoma. Besides, they were instructed in the method of making appointments to recheck in stoma clinic. All the contents were sent to the groups, and the same contents were sent circularly in second half of the month to repeatedly enhance the patients' understanding. ⑤ The team members regularly viewed the chatting contents in the group every day and promptly answered the inquiries about the disease from the patients and their families. If some patient did not send message to the WeChat group for 1 week, the team members should promptly contact the patient by phone to inform him/her of the significance of participating in the group chats and encourage him/her to actively participate in the communication. The intervention cycles in both groups were 1 months

### 2.3. Evaluation Indexes

After intervention, the fasting elbow vein blood (4 mL) was collected from every patient in the two groups and was put into the centrifuge tubes. The centrifuge tubes were placed at 37°C to promote the blood to coagulate. When being coagulated, the blood was centrifuged, and the clear supernatant was blood serum. The blood serum was drawn and subpackaged carefully for reservation. The automatic biochemical analyzer (manufacturer: Puyang City Hukang Medical Equipment Co., Ltd.; model: XR420A.) was adopted to detect the nutrition indicators, including the albumin (ALB), serum prealbumin (PA), and transferrin (TRF).

The immunoturbidimetry was adopted to detect the levels of the immunoglobin A (IgA), immunoglobin M (IgM), and immunoglobin G (IgG) in the serum samples.

The World Health Organization Quality of Life (WHOQOL)-BREF [13] was adopted to assess the living condition of the patients in the two groups after intervention. This questionnaire was the simplified version of World Health Organization Quality of Life (WHOQOL)-100. WHOQOL-BREF was mainly used to see the research objects' feelings about their own living condition, daily activities, and health status. This questionnaire included physiological dimension, psychological dimension, dimension of social relationship, and environment dimension, and the patients were given scores from the 4 dimensions with 5 grades. The total score (28-140 points) was the sum of all the items (28 items), and higher scores indicated better health conditions of the research objects.

The self-rating anxiety scale (SAS) [14] and the self-rating depression scale (SDS) [15] were used to evaluate the psychological state of the two groups after intervention. The cut-off value of SAS was 50 points. According to SAS, the patients with less than 50 points were considered normal, the patients with 50-59 points were considered to suffer from mild anxiety, the patients with 60-69 points moderate anxiety, and the patients with 70 points or more than 70 points severe anxiety. The cut-off value of SDS was 53 points. According to SDS, the patients with less than 53 points were considered normal, the patients with 53-62 points were considered to suffer from mild depression, the patients with 63-72 points moderate depression, and the patients with more than 72 points severe depression.

The complications of the patients in the two groups were recorded and counted. The complications included edema of stoma tissues, stoma stenosis, hernia around the stoma and prolapse of the stoma.

### 2.4. Statistical Treatment

The professional statistical software SPSS26.0 was adopted for data processing and GraphPad Prism 7 (GraphPad Software, San Diego, USA) was used to draw graphs of the data in this study. The count data were tested by *X*^2^ and expressed by (*n* (%)). The measurement data were tested by *t* and expressed by mean ± SD. When *P* < 0.05, the differences were considered statistically significant.

## 3. Results

### 3.1. Clinic Data

There was no remarkable difference in the sex ratio, mean age, pathological type, education level, and other clinic data between the two groups (*P* > 0.05; Table 1).

### 3.2. Nutrition Indicators

After intervention, the various nutrition indicators of the study group were all higher than those of the reference group (*P* < 0.001; Table 2).

### 3.3. Immune Indexes

After intervention, the various immune indexes of the study group were all prominently higher than those of the reference group (*P* < 0.05; Table 3).

### 3.4. WHOQOL-BREF Score

After intervention, the WHOQOL-BREF score of the study group was prominently higher than that of the reference group (*P* < 0.001; Figure 1).

### 3.5. Psychological State

Compared with the reference group, the study group after intervention achieved markedly lower SAS score and SDS score (*P* < 0.001; Figure 2).

### 3.6. Complications

Compared with the reference group, the study group achieved obviously lower total incidence of complications (*P* < 0.05; Table 4).

## 4. Discussion

Rectal cancer is the general name for the malignant tumors occurring in the rectum, and it has multiple pathogenic factors, including environment, heredity, colorectal adenoma, and ulcerative colitis. Low rectal cancer is a common type of rectal cancer [16]. Most patients with low rectal cancer seek medical treatment for the severe ileus and inflammatory edema in the intestinal wall, and colostomy is needed to relieve their clinical symptoms before performing the radical resection of rectal cancer. However, clinical studies [17] have confirmed that the patients with low rectal cancer are likely to have multiple complications after colostomy, which affects patients' postoperative recovery and prolongs their hospitalization time. As a result, their quality of life is greatly reduced. Therefore, it is of great clinical significance to provide good intervention for the patients with low rectal cancer after colostomy.

The growth of tumors often consumes a large amount of nutrients, so the patients' nutritional status may deteriorate. Besides, the rectal cancer, as a common malignant tumor in the digestive system, affects the intake, digestion, and absorption of nutrients because the tumor occurs in the alimentary canal, so the incidence of nutritional risk is significantly higher than that of other malignant tumors [18, 19]. In recent years, there have been more studies about the application of nutritious meal in the critically ill patients, and all the study results have shown that it can improve patients' intestinal function, help the patients to better control their blood glucose, and reduce and prevent bacterial translocation [20]. Therefore, most hospitals take nutritious meal as the first choice of the nutritional support at present because it can reduce the patients' postoperative complications and promote the recovery of the intestinal functionand the scientific meal plan can further enhance the patients' immune function and improve their intestinal barrier function which have been confirmed in the patients with bile duct cancer, colon cancer or other diseases[19, 21]. The Internet, with massive information, sharing characteristic, interactivity, promptness, and the hypertext, has been widely applied in the innovative mode of health education in hospitals. The clinical education and publicity based on the Internet effectively break through the obstacle of the information dissemination and make up for the shortcomings of the traditional health education mode in hospitals. Besides, the combination of the Internet and the clinical education and publicity develops new channels of postoperative health education for patients and improves the work enthusiasm of the medical workers, conducive to building harmonious doctor-patient relationship and enhancing the patients' self-management ability, and the effect of online publicity and education has been confirmed in the application to AIDS patients [22].

However, there is no study on the intervention effects of nutritious meal combined with online publicity and education on the patients with low rectal cancer after colostomy. In this study, a controlled clinical trial was conducted, and 88 patients with low rectal cancer who received the colostomy in our hospital (August 2020-August 2021) were given different postoperative interventions, aiming at providing more evidence-based proofs for these patients. The sera ALB, PA, and TRF are the common indicators directly reflecting the nutritional status of the human body. According to the study results, the various nutrition indicators of the study group after intervention were prominently higher than those of the reference group (*P* < 0.001), indicating that the nutritious meal combined with online publicity and education can greatly promote the nutritional status of the patients with low rectal cancer after colostomy, protect their intestinal mucosa, and speed up the recovery of their intestinal function, so as to provide the nutritious substance the body needed. The reasons are speculated as follows. The various substances contained in the nutritious meal can be absorbed by the body through the venous system, which facilitates synthesizing protein in the digestive tract, regulating metabolism, and protecting liver and kidney function [23]. Besides, such intervention method can effectively improve the intestinal barrier function of the patients with gastrointestinal cancer, thus greatly reducing bacterial translocation and relieving the patients' inflammatory response. In terms of the complication, the total incidence in the study group after intervention was markedly lower than that of the reference group. The reasons are as follows. Nutritious meal can promote the gallbladder contraction and gastrointestinal motility, increasing blood flow in the viscera and decreasing the burden of circulatory system and the complications in other systems. As a result, the patients' metabolism is more suitable for the normal physiological process, which is conducive to their postoperative rehabilitation [24].

## 5. Conclusion

In conclusion, nutritious meal combined with online publicity and education is a reliable method of improving the postoperative nutrition and psychological state of the patients with low rectal cancer after colostomy and has clinical application value. The implementation of this method can reduce the incidence of complications and enhance the patients' immune function. However, the samples selected in this study are too few to draw a conclusion, and it is necessary to conduct the multicenter controlled randomized clinical trial in future to verify the results in this study. Besides, in terms of the follow-up, the short-term follow-up is not enough to effectively evaluate the patients' survival time, so it is necessary to do more high-quality and multicentric studies to confirm the effectiveness of nutritious meal combined with online publicity and education.

## Figures and Tables

**Figure 1:** Comparison of the WHOQOL-BREF score (mean ± SD). Notes: the abscissa referred to the study group and reference group, and the ordinate indicated the WHOQOL-BREF score (points); The WHOQOL-BREF scores of the study group and the reference group were 115.80 ± 9.83 points and 103.05 ± 11.67 points, respectively. ^∗^A remarkable difference in the WHOQOL-BREF score between the two groups (*t* = 5.543, *P* < 0.001).

**Figure 2:** Comparison of the psychological state (mean ± SD). Notes: (a) The comparison of SAS scores between the two groups. In (a), the abscissa referred to the study group and reference group, and the ordinate indicated SAS score (points). The SAS scores of the study group and the reference group were 40.75 ± 7.34 points and 47.61 ± 4.74 points, respectively. ^∗^A remarkable difference in SAS score between the two groups (*t* = 5.208, *P* < 0.001). (b) The comparison of SDS scores between the two groups. In (b), the abscissa referred to study group and reference group and the ordinate indicated SDS score (points). The SDS scores of the study group and the reference group were 40.95 ± 5.30 points and 47.50 ± 5.55 points, respectively. ^∗∗^A remarkable difference in the SDS score between the two groups (*t* = 5.662, *P* < 0.001).

**Table 1:** Comparison of the clinic data.

Item	Study group	Reference group	*X* ^2^/*t*	*P*
Sex (*n* (%))			0.202	0.653
Male/female	28/16	30/14		
Mean age (mean ± SD, years old)	65.59 ± 9.28	65.91 ± 9.73	0.158	0.875
BMI (body mass index, mean ± SD, kg/m^2^)	23.51 ± 2.67	23.29 ± 3.00	0.363	0.717
Smoking history (*n* (%))			0.188	0.665
Yes	19 (43.18)	17 (38.64)		
No	25 (56.82)	27 (61.36)		
Drinking history (*n* (%))			0.182	0.669
Yes	22 (50.00)	20 (45.45)		
No	22 (50.00)	24 (5.55)		
Pathological type (*n* (%))				
Medium differentiated adenocarcinoma	31 (70.45)	31 (70.45)	0.000	1.000
Adenocarcinoma	3 (6.82)	4 (9.09)	0.075	0.784
Medium-low differentiated adenocarcinoma	2 (4.55)	3 (6.82)	0.212	0.645
Mucinous cancer	2 (4.55)	1 (2.27)	0.345	0.557
Highly differentiated adenocarcinoma	1 (2.27)	0 (0.00)	1.012	0.315
Signet-ring cell carcinoma	1 (2.27)	0 (0.00)	1.012	0.315
Poorly differentiated adenocarcinoma	1 (2.27)	1 (2.27)	0.000	1.000
Poorly differentiated squamous cell carcinoma	0 (0.00)	1 (2.27)	1.012	0.315
Villous adenoma	0 (0.00)	1 (2.27)	1.012	0.315
High-grade prostatic intraepithelial neoplasia	1 (2.27)	0 (0.00)	1.012	0.315
Highly differentiated adenocarcinoma	2 (4.55)	2 (4.55)	0.000	1.000
Underlying diseases (*n* (%))				
Hypertension	6 (13.64)	8 (18.18)	0.340	0.560
Diabetes	3 (6.82)	5 (11.36)	0.550	0.458
Atrial fibrillation	4 (9.09)	3 (6.82)	0.155	0.694
Chronic gastritis	5 (11.36)	4 (9.09)	0.124	0.725
Hyperthyroidism	2 (4.55)	3 (6.82)	0.212	0.645
Nephrolithiasis	3 (6.82)	2 (4.55)	0.212	0.645
Coronary atherosclerotic heart disease	1 (2.27)	0 (0.00)	1.012	0.315
Types of stoma (*n* (%))				
Transverse colostomy	2 (4.55)	0 (0.00)	2.047	0.153
Colostomy of descending colon	12 (27.27)	9 (20.45)	0.563	0.453
Single-cavity sigmoidostomy	15 (34.09)	21 (47.73)	1.692	0.193
Proximal sigmoidostomy	2 (4.55)	2 (4.55)	0.000	1.000
Sigmoidostomy	13 (29.55)	11 (25.00)	0.229	0.632
Double-cavity sigmoidostomy	0 (0.00)	1 (2.27)	1.012	0.315
Education level (*n* (%))				
Bachelor degree and higher	2 (4.55)	3 (6.82)	0.212	0.645
Junior college	3 (6.82)	2 (4.55)	0.212	0.645
Senior high school	7 (15.91)	6 (13.64)	0.090	0.764
Middle school	13 (29.55)	11 (25.00)	0.229	0.632
Primary school	17 (38.64)	15 (34.09)	0.196	0.658
Illiteracy	2 (4.55%)	7 (15.91%)	3.094	0.079
Place of residence (*n* (%))			0.183	0.669
Urban areas	19 (43.18%)	21 (47.73%)		
Rural areas	25 (56.82%)	23 (52.27%)		

**Table 2:** Comparison of the nutrition indicators (mean ± SD).

Group	*n*	ALB (g·L^−1^)	PA (mg·L^−1^)	TRF (g·L^−1^)
Study group	44	38.55 ± 4.22	153.19 ± 3.99	162.92 ± 6.88
Reference group	44	35.24 ± 2.20	138.50 ± 1.95	138.45 ± 6.61
*t*		4.614	21.941	17.013
*P*		<0.001	<0.001	<0.001

**Table 3:** Comparison of the immune indexes (mean ± SD, mg/L).

Group	*n*	IgA	IgM	IgG
Study group	44	145.10 ± 6.27	158.38 ± 6.45	145.48 ± 4.06
Reference group	44	140.66 ± 3.95	146.26 ± 4.04	132.92 ± 2.47
*t*		3.974	10.563	17.531
*P*		<0.05	<0.001	<0.001

**Table 4:** Comparison of the complications (*n* (%)).

Group	n	Edema of stoma tissues	Stoma stenosis	Hernia around the stoma	Prolapse of the stoma	Total incidence
Study group	44	0(0.00)	1(2.27)	0(0.00)	1(2.27)	4.55%(2/44)
Reference group	44	1(2.27)	2(4.55)	2(4.55)	3(6.82)	18.18%(8/44)
*X* ^2^						4.062
P						<0.05

## Data Availability

Data to support the findings of this study is available on reasonable request from the corresponding author.
